RETRACTED

# Effects of Different Doses of Clopidogrel plus Early Rehabilitation Therapy on Motor Function and Inflammatory Factors in Patients with Ischemic Stroke

**DOI:** 10.1155/2022/9692382

**Published:** 2022-06-14

**Authors:** Zhuolin Zhao, Ying Ma, Qin Liu, Ling Jiang, Huimin Shu, Daofeng Chen, Jiao Wu

**Affiliations:** ^1^Department of Neurology, The Second People's Hospital of Yibin, Yibin, China; ^2^Department of Neurology, North Sichuan Medical College, Nanchong, China; ^3^Department of Neurosurgery, The Second People's Hospital of Yibin, Yibin, China

## Abstract

This prospective randomized controlled study was intended to assess the effects of different doses of clopidogrel plus early rehabilitation therapy on motor function and inflammatory factors in patients with ischemic stroke. Between August 2018 and October 2020, 90 cases of ischemic stroke treated in the Second People's Hospital of Yibin were randomized at a ratio of 1 : 1 to receive either oral 50 mg/d clopidogrel plus early rehabilitation therapy (low-dose group) or oral 75 mg/d clopidogrel plus early rehabilitation therapy (high-dose group), with 45 cases in each group. The outcome measures including the Barthel Index (BI), National Institutes of Health Stroke Scale (NIHSS), Fugl-Meyer simplified scale, hypersensitive C-reactive protein (hs-CRP), interleukin-6 (IL-6), tumor necrosis factor-*α* (TNF-*α*), and occurrence of adverse events were collected. After treatment, the high-dose group had higher BI results than the low-dose group. All eligible patients showed significantly declined NIHSS scores, and the high-dose group had markedly lower results (*P* < 0.05). After treatment, the Fugl-Meyer scores of both upper and lower extremities of the high-dose group were significantly higher than those in the low-dose group. The high-dose group achieved a greater decrease in inflammatory factor levels after treatment versus the low-dose group. The two groups showed a similar incidence of adverse events. High-dose clopidogrel plus early rehabilitation outperforms the low-dose treatment for patients with ischemic stroke by effectively mitigating the inflammatory response in the body, promoting the restoration of neurological function, improving the level of motor function, and enhancing the patient's quality of life, with manageable safety.

## 1. Introduction

Ischemic stroke is a common cerebrovascular disease with pathogenesis associated with the formation of thrombus after atherosclerosis, and its prevalence is higher in the elderly population. Ischemic stroke is characterized by rapid onset and progression, easy recurrence, and high disability and mortality rate [1, 2]. Relevant studies have reported that patients may experience symptoms such as syncope after the onset of ischemic stroke as a result of blood circulation disorders in the brain and vascular embolism [3, 4]. Despite a relatively decreased mortality of ischemic stroke, thanks to the advancement of medical technology, 3/4 of surviving patients still suffer from varying degrees of compromised life quality [5]. Thus, timely and effective rehabilitation may facilitate the recovery of neurological function, improve the quality of life, and ameliorate the prognosis of patients with ischemic stroke [6]. According to traditional Chinese medicine (TCM), the pathogenesis of ischemic stroke is complex and is mainly associated with blood stasis, deficiency of qi and blood, and the accumulation of fire, which result in insufficient blood supply to the brain and cerebral hemorrhage and then lead to brain blockage and impaired body function. Therefore, clinical nursing should pay attention to the activity of muscles and collaterals to enhance blood circulation and avoid stasis. TCM treatment of ischemic stroke mainly relies on rehabilitation exercises and nursing through interventions related to psychological management, acupressure, health education, and rehabilitation training to improve patients' treatment compliance, restore their limb functions, and lower the disability rate [7].

RETRACTED

Prior research has shown significantly elevated expression levels of hypersensitive C-reactive protein (hs-CRP), interleukin-6 (IL-6), and tumor necrosis factor (TNF-*α*) in patients with ischemic stroke [8]. The clinical treatment of acute ischemic stroke mainly involves thrombolysis, antiplatelet, lipid-lowering, and improvement of the cerebral circulation to restore blood perfusion to brain tissue. Clopidogrel is an adenosine diphosphate (ADP) receptor antagonist that hinders platelet aggregation by binding to the platelet membrane surface ADP receptor and inhibiting its expression to alleviate the inflammatory response [9]. However, clinical consensus on the use of either low-dose or high-dose clopidogrel treatment has not yet been established. Accordingly, this study analyzed and investigated the effects of low-dose versus high-dose clopidogrel plus early rehabilitation therapy on motor function and inflammatory factor levels in patients with ischemic stroke.

## 2. Materials and Methods

### 2.1. Baseline Data

It was a prospective randomized controlled study that enrolled 90 cases of ischemic stroke treated in the Second People's Hospital of Yibin from August 2018 to October 2020. All enrollments were randomized at a ratio of 1 : 1 to receive either oral 50 mg/d clopidogrel plus early rehabilitation therapy (low-dose group) or oral 75 mg/d clopidogrel plus early rehabilitation therapy (high-dose group), with 45 cases in each group. The protocol of the study was ethically approved by the Ethical Committee of the Second People's Hospital of Yibin (no. 2018-E12/839).

RETRACTED

### 2.2. Inclusion and Exclusion Criteria

Inclusion criteria: patients who met the diagnostic criteria in the Chinese Ischemic Stroke Diagnostic and Treatment Guidelines 2018 and the diagnosis was confirmed by MRI or CT scan; with medication; without serious mental illness, with normal cognition to effectively cooperate with treatment; and who provided written informed consent were included. Exclusion criteria: patients with contraindications to drug interventions in the study; with serious hematologic, autoimmune, and hepatic and renal system diseases; with serious complications such as arrhythmias, heart failure, and shock; and with serious mental illness and cognitive impairment were excluded.

### 2.3. Methods

Medication: in both groups, 10 mL of 0.9% sodium chloride solution + 10 *μ*g of prostaglandin were administered through injection daily to improve cerebral microcirculation, and 0.5 mg of methylcobalamin was administered orally daily to nourish nerves. On this basis, the low-dose group received oral 50 mg of clopidogrel (Shenzhen Xinlitai Pharmaceutical Co., Ltd., approval no. H20000542) daily, and the high-dose group received 75 mg of clopidogrel daily.

Early rehabilitation: the early rehabilitation therapy was carried out after the patient's vital signs were stabilized. (1) The patients were instructed and assisted to perform correct limb placement. The patient's shoulder joint was bent forward, a thick and soft pillow was placed on the chest with the upper extremity of the affected side on the pillow, and the elbow and wrist of the affected side were extended with the back of the hand upward. The knee and hip joints on the healthy side were slightly flexed, and a soft pillow was placed on the healthy lower limb with the affected lower limb flexed and placed on the pillow. The patients were assisted to perform the appropriate placement of the affected limbs. The patient's upper extremity on the affected side was abducted at 90°, followed by extension of the elbow joint, a forward extension of the scapula, and the dorsal extension of the wrist joint, with the palm upward. The upper extremity of the patient's healthy side was placed on the trunk. The knee joint of the affected lower extremity was slightly flexed, the hip joint was extended, and a soft pillow was placed on the back and the affected lower extremity, followed by the lower extremity of the patient's healthy side flexed and placed on the pillow. (2) Motor imagery: the patient was assisted to adopt a supine position and was guided to imagine a comfortable state and intermittently perform motor imagery (such as grasping a ping-pong ball or a wooden peg) to improve the function of the finger and wrist. (3) Motor therapy: active and passive training of the patient's affected limb was performed using the Bobath method. Passive movements were performed on the joints of the patient's whole body during bed mobility. The ten fingers of the patient's hands were crossed, and the thumb of the patient's healthy side was placed under the affected thumb and gently abducted outward, using the healthy limb to guide the affected limb in performing lifting movements. (4) Occupational therapy: the patient was assisted to perform daily activities such as washing, eating, changing clothes, and using the toilet as independently as possible. The patient's family members were also instructed to help the patient restore their self-care ability. (5) TCM-based acupoint massage: the patient received acupoint massage for 10 min, twice daily (in the morning and in the evening). After discharge from the hospital, the massage was performed by the patient's families or healthcare providers who received massage instructions and guidance from professional nursing staff in the hospital. Massage acupoints mainly include Baihui, Taihong, and Hegu acupoints.

RETRACTED

### 2.4. Clinical Outcomes

1. Barthel Index (BI): the total score of BI is 100 points, and the assessments were performed on daily feeding, dressing, bathing, bowel control, walking, toileting, going up and down stairs, and bed and chair transfer of the patients. The higher the score, the better the self-care ability.
2. National Institutes of Health Stroke Scale (NIHSS): the NIHSS score ranges from 0 to 42 points, and the assessments were performed on consciousness, limb movement, temperature, ataxia, visual field, and gaze. The higher the score, the higher the degree of neurological impairment.
3. Fugl-Meyer simplified scale: the Fugl-Meyer simplified scale was used to score the recovery of upper and lower limb motor function in both groups before and after treatment. The total upper extremity motor function score was 66 points, and the total lower extremity motor function score was 34 points. The higher the Fugl-Meyer score, the better the recovery of motor function of upper and lower limbs.
4. Inflammatory factor levels: 3 mL of venous blood was collected from patients before and after treatment, respectively. The blood samples were added with hs-CRP, TNF-*α*, and IL-6 monoclonal antibodies and irrigated with PBS solution for 5 min. 5 mL of sheep anti-Human primary antibody was added (1 : 500), left overnight at 4°C, rinsed 3 times with PBS buffer for 5 min each time, followed by the addition of 2 mL of anti-mouse secondary antibodies (1 : 1000), left at room temperature for 2 h, and rinsed with PBS solution for 5 min. Then, horseradish peroxidase was used for color development and a termination solution was used to stop the color reaction. The OD value was measured at 450 nm.
5. Adverse events: adverse events include increased eosinophilia, abnormal liver function, cerebral hemorrhage, and gastrointestinal bleeding.

RETRACTED

### 2.5. Statistical Analysis

SPSS 20.0 was used for data analyses, and GraphPad Prism 8 was used to visualize the data into required graphics. The measurement data are expressed as (mean ± standard deviation) and analyzed using the independent samples *t*-test. The count data are expressed as the number of cases (rate) and analyzed using the chi-square test. Statistically significant results were defined as *P* < 0.05.

## 3. Results

### 3.1. Comparison of General Data

In the low-dose group, there were 23 males and 22 females, aged 42–80 years, mean age of 60.31 ± 5.49 years, 12 patients with left-sided hemiparesis, 20 patients with right-sided hemiparesis, and 13 patients with bilateral hemiparesis. In the high-dose group, there were 21 males and 24 females, aged 42–81 years, mean age of 60.58 ± 5.36 years, 14 patients with left-sided hemiparesis, 17 patients with right-sided hemiparesis, and 14 patients with bilateral hemiparesis. The baseline characteristics of the two groups were comparable (*P* > 0.05) (Table 1).

### 3.2. Comparison of BI

Before treatment, the BI in the low-dose group was 50.27 ± 5.71 points and 50.35 ± 5.59 points in the high-dose group, and intergroup differences were not significant (*P* > 0.05). After treatment, the BI was 69.41 ± 6.82 points in the low-dose group and 79.62 ± 7.51 points in the high-dose group, with higher BI results observed in the high-dose group (*P* < 0.05) (Figure 1).

### 3.3. Comparison of NIHSS Scores

Before treatment, the NIHSS was 11.62 ± 2.11 points in the low-dose group and 11.55 ± 1.96 points in the high-dose group, without significant intergroup differences (*P* > 0.05). After treatment, the NIHSS was 8.46 ± 1.32 points in the low-dose group and 6.62 ± 1.17 points in the high-dose group, and the high-dose group had lower NIHSS results (*P* < 0.05) (Figure 2).

### 3.4. Comparison of Fugl-Meyer Scores

The Fugl-Meyer score of the upper extremity in the low-dose group was 20.12 ± 10.06 points before treatment and 28.44 ± 9.61 points after treatment, and the Fugl-Meyer score of the lower extremity was 17.21 ± 10.35 points before treatment and 25.74 ± 8.39 points after treatment. The Fugl-Meyer scores of the upper extremity in the high-dose group were 20.23 ± 10.12 points before treatment and 42.57 ± 10.20 points after treatment, and the Fugl-Meyer scores of the lower extremity were 16.97 ± 10.19 points before treatment and 32.57 ± 6.88 points after treatment. After treatment, the Fugl-Meyer scores of both upper and lower extremities of the patients in the high-dose group were significantly higher than those in the low-dose group (*P* < 0.05) (Table 2).

RETRACTED

### 3.5. Comparison of Inflammatory Factors

There were no significant differences in the levels of hs-CRP, TNF-*α*, and IL-6 between the two groups of patients before treatment (*P* > 0.05). After treatment, hs-CRP was 9.08 ± 1.65 mg/L, TNF-*α* was 55.21 ± 12.14 ng/L, and IL-6 was 9.35 ± 2.15 pg/ml in the low-dose group, and hs-CRP was 7.34 ± 1.72 mg/L, TNF-*α* was 46.16 ± 12.57 ng/L, and IL-6 was 7.94 ± 2.22 pg/ml in the high-dose group. The levels of inflammatory factors decreased in both groups, with lower results observed in the high-dose group versus the low-dose group (*P* < 0.05) (Table 3).

### 3.6. Comparison of Adverse Events

In the low-dose group, there was 1 case of increased eosinophils, 1 case of abnormal liver function, 1 case of cerebral hemorrhage, and 2 cases of gastrointestinal bleeding, with an adverse events rate of 11.11% (5/45). In the high-dose group, there were 2 cases of abnormal liver function, 1 case of cerebral hemorrhage, and 1 case of gastrointestinal bleeding, with an adverse events rate of 8.89% (4/45). The two groups showed a similar incidence of adverse events (*P* > 0.05) (Table 4).

## 4. Discussion

In the pathogenesis of ischemic stroke, the rupture of atherosclerotic plaque induces local hemodynamic abnormalities in brain tissue and increases blood viscosity, resulting in hypoxia and ischemic necrosis of the brain tissue. Improper or ineffective treatment may lead to serious neurological sequelae that threaten the life of patients [10–12]. Clopidogrel is a commonly used drug for ischemic stroke and is an inactive precursor drug that binds ADP receptors on the platelet membrane surface, preventing the glycoprotein GPIIb/IIIa receptors from binding to fibrinogen and antagonizing platelet aggregation. Clopidogrel blocks ADP receptors, inhibits the release of cytokines from platelets, avoids macrophage activation, activates the CD40-CD40 L signaling pathway, and mitigates the inflammatory response. It inhibits the release of interleukins and other inflammatory transmitters, attenuates endothelial damage, lowers serum CRP levels, suppresses the inflammatory response, and relieves the patient's cerebral hypoxia and ischemia to protect neurological function. The results of the present study showed that after treatment, NIHSS scores were significantly reduced in both groups, with a lower level in the high-dose group than in the low-dose group, suggesting that high-dose clopidogrel was more effective in mitigating neurological impairment. The levels of inflammatory factors decreased in both groups, with lower results observed in the high-dose group versus the low-dose group. High-dose clopidogrel better promotes reperfusion in the ischemic penumbra, shrinks the infarct volume, increases neuronal activity, attenuates the degree of cerebral ischemic injury, alleviates the inflammatory response of the body, increases the blood flow supply to the ischemic brain, facilitates the improvement of prognosis, and improves the ability of patients in daily life, which is consistent with the findings by Liang Hua [13–16]. It has been reported that patients with ischemic stroke may experience abnormal motor function such as hemiparesis after treatment, which dramatically compromises their daily life. Hence, the improvement of the prognosis of stroke patients' motor function and their quality of life remains a key issue in the rehabilitation of patients to be addressed. In recent years, the standardized early rehabilitation treatment for ischemic stroke patients efficiently boosts the effectiveness of their rehabilitation in clinical practice. In early rehabilitation, the patient's scapular position is effectively managed to prevent the occurrence of myospasm, and the upper and lower extremities are extended or flexed to reduce the incidence of hemiplegic limb complications. Motor imagery strengthens the brain-to-muscle movement pattern and accelerates the recovery of the motor reflex arc. In addition, proper motor training for patients significantly improves their abnormal motor patterns, attenuates their muscle spasticity, and promotes their early recovery [17–21]. The results of the present study showed that after treatment, the high-dose group showed higher BI results versus the low-dose group (*P* < 0.05), which indicated that high-dose clopidogrel plus early rehabilitation significantly improved patients' self-care ability. After treatment, the higher dose group had higher Fugl-Meyer scores in both upper and lower extremities than the low-dose group, indicating that high-dose clopidogrel plus early rehabilitation therapy was more effective in improving the motor function of patients. Furthermore, the absence of differences in the adverse events between the two groups suggests a manageable safety profile of the high-dose therapy of clopidogrel.

RETRACTED

## 5. Conclusion

High-dose clopidogrel plus early rehabilitation outperforms the low-dose treatment for patients with ischemic stroke by effectively mitigating the inflammatory response in the body, promoting the recovery of neurological function, improving the level of motor function, and enhancing the patient's quality of life, with manageable safety.

## Figures and Tables

**Figure 1:** Comparison of BI.

**Figure 2:** Comparison of NIHSS scores.

**Table 1:** Comparison of baseline data.

	Low-dose group (*n* = 45)	High-dose group (*n* = 45)	*t*/*χ*^2^	*P*
Gender (male/female)	23/22	21/24	0.178	0.673
Age (year)	60.31 ± 5.49	60.58 ± 5.36	0.233	0.816
Lesion position			0.434	0.805
Left-sided	12	14		
Right-sided	20	17		
Bilateral	13	14		

**Table 2:** Comparison of Fugl-Meyer scores ($\bar{x}$ ± *s*).

Groups	*n*	Upper extremity Fugl-Meyer scores		Lower extremity Fugl-Meyer scores	
		Before treatment	After treatment	Before treatment	After treatment
Low-dose group	45	20.12 ± 10.06	28.44 ± 9.61	17.21 ± 10.35	25.74 ± 8.39
High-dose group	45	20.23 ± 10.12	42.57 ± 10.20	16.97 ± 10.19	32.57 ± 6.88
*t*	—	0.052	6.764	0.111	4.223
*P*	—	0.959	<0.001	0.912	<0.001

**Table 3:** Comparison of inflammatory factor ($\bar{x}$ ± *s*).

Groups	*n*	Hs-CRP (mg/L)		TNF-*α* (ng/L)		IL-6 (pg/ml)	
		Before	After	Before	After	Before	After
Low-dose group	45	12.37 ± 2.72	9.08 ± 1.65	61.34 ± 12.98	55.21 ± 12.14	15.87 ± 3.84	9.35 ± 2.15
High-dose group	45	12.35 ± 2.74	7.34 ± 1.72	61.51 ± 13.15	46.16 ± 12.57	15.93 ± 3.67	7.94 ± 2.22
*t*	—	0.035	4.897	0.062	3.474	0.076	3.061
*P*	—	0.972	<0.001	0.951	0.001	0.94	0.003

**Table 4:** Comparison of adverse events (*n* (%)).

	*n*	Increased eosinophils	Abnormal liver function	Cerebral hemorrhage	Gastrointestinal bleeding	Total incidence
Low-dose group	45	1	1	1	2	5 (11.11%)
High-dose group	45	0	2	1	1	4 (8.99%)
*t*	—					0.123
*P*	—					0.725

## Data Availability

The datasets used during the present study are available from the corresponding author upon request.
